# Predictive Factors for Late-Onset Neurological Deficits in Patients with Posttuberculous Thoracic Kyphosis

**DOI:** 10.1155/2022/8555924

**Published:** 2022-09-07

**Authors:** Jianquan Zhao, Zhuyun Cai, Yicheng Meng, Xuhui Zhou, Heng Jiang

**Affiliations:** Department of Orthopedic Surgery, Changzheng Hospital, Second Military Medical University, Shanghai 200003, China

## Abstract

**Background:**

Patients with severe posttuberculous (TB) kyphosis might suffer from late-onset neurological deficits, and surgical correction may improve neurological function. However, there is a lack of predictive factors for neurological function in these patients.

**Objective:**

This study was aimed at identifying the risk factors for late-onset neurological deficits in spinal TB patients at initial and final assessments.

**Methods:**

Seventy-eight patients with severe kyphosis caused by old thoracic tuberculosis were retrospectively analyzed. Patients with active spinal TB and other spinal diseases were excluded from the analysis. The kyphosis Cobb angle, sagittal deformity angular ratio (S-DAR), and level of apex were measured and calculated on X-ray. The spinal cord cross-sectional area ratio (CSAR), spinal cord sagittal diameter ratio (SDR), and spinal cord angle (SCA) were measured on preoperative T2-weighted magnetic resonance imaging (MRI). According to the American Spinal Injury Association (ASIA) Impairment Scale (AIS) at the time of admission, the patients were divided into the symptomatic group (*N* = 60 patients, AIS grades A to D) and the asymptomatic group (*N* = 18 patients, AIS grade E). All of the symptomatic patients underwent surgery, and the patients from both groups had at least 2 years of follow-up. Relationships among the radiological parameters and initial and final AIS grades were evaluated via univariate and multivariate analyses.

**Results:**

The mean duration of kyphotic deformity was 37.4 years in the symptomatic group. There were no significant differences between the two groups in terms of CSAR, kyphosis Cobb angle, S-DAR, level of apex, or the segments that were involved. Patients from the symptomatic group exhibited significantly greater SDR and smaller SCA than those from the asymptomatic group (*p* < 0.01 and *p* < 0.01, respectively). The multivariate logistic regression identified SDR and SCA as independent factors influencing the likelihood of spinal cord injury at the initial and final assessments.

**Conclusions:**

Severe posttuberculous kyphosis may lead to significant neurological symptoms many years following the initial treatment. The predictive factors for late-onset neurological deficits include larger SDR and smaller SCA.

## 1. Introduction

Spinal tuberculosis (TB) often involves the thoracic and lumbar segments and is a major cause of kyphotic deformities [1]. Although chemotherapy has resulted in TB being a curable disease [2], the structure of the spine is destroyed after TB infection, thus resulting in severe kyphosis (Pott's deformity), spinal instability, and the tendency to develop nonunion [1]. Severe kyphotic deformities can lead to severe appearance and psychological problems in patients. In addition, late-onset neurological deficits may occur after many years in a healed TB, which may be due to spinal cord compression or traction caused by bulging of the central vertebral bone in the angular kyphosis into the spinal canal, as well as due to the proliferation of fibrous tissue in the spinal canal and the excessive traction of the spinal cord caused by kyphosis [3]. Therefore, it is of great significance to predict or prevent the occurrence of delayed neurological dysfunction in patients with healed TB.

To our knowledge, there are few studies that have examined radiological parameters in healed spinal TB to define the risk factors for late-onset neurological deficits or to predict the prognoses of the neurological outcomes after surgery. Clinical studies have demonstrated that risk factors, including thoracic kyphosis, cord edema, and canal encroachment, can predict neurological deficits in patients with active spinal TB [4–7]. However, the previous literature has limited information on effective evaluation methods or indicators for evaluating and predicting changes in neurological function [8], which may have a direct guiding role in the treatment and prognosis of the disease, especially in deciding the timing of surgery.

Therefore, the purpose of this study was to assess the risk factors for late-onset neurological deficits in patients with severe posttuberculous thoracic kyphosis at the initial and final assessments.

## 2. Methods

### 2.1. Participants

The details of patients with Pott's deformity (apex levels T1 to T12, inclusive) presented at Shanghai Changzheng hospital spinal deformity center between 2013 and 2020 were retrospectively obtained. Research ethics and institutional review boards approved the study. Patients were included if they were older than 18 years old, had a severe kyphotic deformity of at least 80° with an apex in the thoracic regions, and had complete imaging data (including full body X-ray and full-spine magnetic resonance imaging (MRI) scans). For patients without surgery, the diagnosis of spinal TB was based on the laboratory tests (such as the Mantoux test, the purified protein derivative (PPD), or the tuberculosis skin test (TST)) and imaging. For operated patients, tissue tests (including culture, histopathology, and polymerase chain reaction (PCR) tests) were also used for the diagnoses. Patients with active diseases, early-onset neurological deficits, cervical or sacral TB, and other severe comorbidities (such as severe restrictive ventilatory disorder) were excluded. Patients with a histological diagnosis of other infections, thoracic kyphosis caused by other causes, or low-quality radiological images that were difficult to accurately measure were also excluded.

Demographic data, including age, sex, duration of kyphosis, and anti-TB therapy, were obtained. The American Spinal Injury Association (ASIA) Impairment Scale (AIS) grades were used for the assessment at the initial presentation and rehabilitation discharge. Patients were divided into the symptomatic group (AIS grades A to D) and the asymptomatic group (AIS grade E).

All of the symptomatic patients who received surgery had a first stage of halo gravity traction, with an average time of 3.2 ± 1.4 months. The second stage of treatment included posterior decompression and stabilization via vertebral column resection (VCR) by one senior spinal surgeon (XHZ) [9]. Motor-evoked potentials (MEPs) and somatosensory evoked potentials (SSEPs) were routinely monitored and recorded during the surgeries. In addition, intraoperative neuromonitoring events were recognized as a decrease in SSEPs of at least 50% amplitude and/or a 10% increase in latency and/or a sustained increase in threshold intensity of at least 100 V for the MEPs [10]. Intraoperative data, including estimated blood loss and operation time, were collected. All of the patients were discharged 14 days after surgery and wore braces for 3 months.

### 2.2. Radiographic Data

Full-spine anteroposterior and lateral radiographs and full-spine MRI were collected for each patient at the initial presentation. For patients undergoing surgery, full-spine anteroposterior and lateral radiographs were also performed at the final follow-up for postoperative kyphosis Cobb angle measurements. The following quantitative measures were performed by using the Picture Archiving and Communication Systems (PACS) system and ImageJ (National Institutes of Health). The angle of kyphotic deformity was determined by using the Cobb angle method as the angle between the upper border of the upper normal vertebrae and the lower border of the lower normal vertebrae [11]. The sagittal deformity angular ratio (S-DAR) was calculated as the Cobb angle of the sagittal curve divided by the number of vertebrae involved in the curve [12]. Additionally, the spinal cord cross-sectional area ratio (CSAR) was calculated by using the following formula: the average of the spinal cord cross-sectional area (CSA) – spinal spinal cord CSA at the apex level/the average of spinal cord CSA ^∗^ 100. The average spinal cord CSA was calculated by taking the average spinal cord CSA of the proximal and distal vertebrae to the diseased segment [13]. The spinal cord sagittal diameter ratio (SDR) was calculated by using the following formula: the average sagittal diameter (SD) of the spinal cord – the SD of the spinal cord at the apex level/the average SD of the spinal cord ^∗^ 100. The average SD of the spinal cord was calculated by taking the average spinal cord SD of the proximal and distal vertebrae to the diseased segment. Moreover, the spinal cord angle (SCA) was defined by the angle formed by two lines that connected the midpoint of the spinal cord at the apex level and the midpoint of the spinal cord at the level of the upper and lower endplates of the destroyed and fused segments before surgery (Figures 1 and 2). The CSAR, SDR, and SCA were measured by 2 independent observers, and the mean value of the 2 measurements was calculated.

### 2.3. Statistical Analysis

Intraclass correlation coefficients, which were calculated by using 2-way mixed intraclass correlation coefficient models (3, *k*), were used for the intrarater and interrater reliability of each observer's measurements. Two-tailed *t*-tests were used for the comparisons between the parametric datasets, and the chi-square test, the Mann–Whitney *U* test (2-tailed), or the Kruskal–Wallis test with a post hoc analysis (the Dunn test) was performed for the comparisons between nonparametric data. Univariate analysis was performed to assess the relationship between independent variables and the presence of spinal cord injury (AIS grades A to D) at the initial and final assessments or regarding no improvement of neurological function after surgery. For the spinal cord cross-sectional area ratio, spinal cord angle, and ratio of sagittal diameter of the spinal cord, ORs were calculated on the basis of having a poor outcome (AIS grades A to D) if compromise was greater than the mean of each group [14]. Variables with a *p* value of < 0.2 in the univariate analysis were chosen for inclusion in a stepwise multivariate logistic model for each binary outcome. Significance was set at *p* < 0.05, and data are presented as the mean and the standard deviation, unless otherwise stated.

## 3. Results

The mean age (and standard deviation) of patients was 45.9 ± 15.8 years, and 67% of patients were male (*n* = 52 patients) (Table 1). The mean duration of kyphotic deformity was 32.4 ± 12.6 years, and 86% of the patients had a history of anti-TB chemotherapy. Additionally, T5 to T8 vertebral levels were the most common levels of the apex (*n* = 43 (55%)). The mean number of segments involved was 6.5 ± 7.6.

Neurological functional change was assessed via the change in AIS grade from the initial assessment (first presentation) to the final assessment (at least 2-year follow-up). Three patients (5%) were classified as AIS grade A at the first visit in the symptomatic group (Table 2, Figure 3). Thirty-five patients in the symptomatic group (58%) showed no change in AIS grade (Table 3). Twenty-one (35%) patients improved AIS grade 1, and 4 (7%) patients improved AIS grade 2 (Table 3).

The mean intraclass correlation coefficients of intrarater reliability were 0.94 ± 0.03, 0.94 ± 0.03, and 0.96 ± 0.03 for the spinal cord cross-sectional area ratio, spinal cord angle, and spinal cord sagittal diameter ratio, respectively. Interrater reliability is shown in Table 4.

We then analyzed the imaging measurement data between the two groups. Patients from the symptomatic group (AIS grades A-D, Figure 4) showed a significantly greater spinal cord sagittal diameter ratio and smaller spinal cord angle than those patients from the asymptomatic group (AIS grade E) (*p* < 0.01 and *p* < 0.01, respectively, Table 5). No significant difference was found in terms of spinal cord cross-sectional area ratio, preoperative sagittal Cobb angle, S-DAR, the involved segments, spinal cord signal change, or levels of apex.

Three independent variables were identified to be associated with patients having spinal cord injury (AIS grades A-D) at the initial and final assessments (Table 6) in the univariate analysis. The spinal cord sagittal diameter ratio and spinal cord angle were identified as being independent factors for the likelihood of spinal cord injury at the initial assessment (OR: 13.56 (95% CI: 3.21-88.43), *p* < 0.01; OR: 8.31 (95% CI: 1.44-32.32), *p* < 0.01, respectively) in the multivariate logistic regression analysis. The spinal cord sagittal diameter ratio and spinal cord angle were identified as being independent factors for the likelihood of spinal cord injury at the final assessment (OR: 8.22 (95% CI: 1.98-43.28), *p* < 0.01; OR: 5.44 (95% CI: 1.10-17.43), *p* < 0.01, respectively).

The spinal cord cross-sectional area ratio and spinal cord angle were identified as being independent factors associated with no improvement in neurological function in the univariate analysis. None of these variables had a significant association with outcomes (*p* > 0.05) in the multivariate logistic regression analysis.

## 4. Discussion

Our study demonstrated that an increased spinal cord sagittal diameter ratio and decreased spinal cord angle were associated with the presence of late-onset neurological deficits in spinal TB, both at the first presentation and at the postoperative follow-up.

Most patients with spinal tuberculosis develop kyphotic deformities in childhood but may still suffer from neurological deterioration many years after the disease is healed [15]. Hsu et al. reported of delayed paraplegia at an average of 18 years after the initial onset of symptoms [16]. Furthermore, Wong et al. reported that approximately 67% of patients presented with late neurological deterioration at a mean of 26 years after the initial drug treatment, and the majority of the deteriorations were caused by healed disease, which leads to worsened results of surgery [17]. In our study, we observed a mean time of 32.4 (6-57) years from the time of the diagnosis of thoracic tuberculosis to the development of delayed neurological dysfunction.

Nerve injury during the quiescence period of posttubercular kyphosis may be caused by direct cord compression by bony structures in front of the spinal canal due to fibrous hyperplasia and the thickening of the epidural granulation tissue or the gradual progression of kyphosis [18]. However, the relationship between kyphotic deformities and the progression of neurological impairment is not yet clear, and there is insufficient evidence in the literature to support the idea that the correction of deformities can prevent neurological degeneration. In our study, we found no association between preoperative kyphosis and spinal cord injury at either the initial or the final assessments.

For patients with thoracic Pott's deformity, there is a lack of effective assessments for predicting the risk of progression of neurological symptoms. In our study, we found that a spinal cord cross-sectional area ratio in excess of 45% showed only a weak association with the development of spinal cord injury either at the first visit or at the final assessment. More importantly, a spinal cord sagittal diameter ratio greater than 47%, which directly reflected the degree of the spinal cord being squeezed or stretched in the sagittal plane, was associated with a greater than tenfold increased likelihood of neurological deficits at first presentation. Although some studies have shown that larger canal encroachment could significantly predict neurological deficits in patients with spine active TB [7], our study indicated that the spinal cord sagittal diameter ratio may be more accurate and useful for predicting late-onset neurological deficits in patients in the quiescent phase of infection.

The relationship between the spinal cord angle and spinal cord injury suggested that traction may be a major cause of injury in cases of thoracic Pott's deformity. The incomplete fusion of the kyphotic deformity and the presence of necrotic cheese tissue were always noted during the operation for patients with neurological symptoms. The appearance of neurological symptoms may also be related to the instability of the deformed apex vertebrae. Therefore, the spinal cord angle (instead of the Cobb angle) may help to detect the early dysfunction of the spinal cord in kyphotic deformities. However, we were unable to identify any relationship between spinal cord angle or spinal cord sagittal diameter ratio and improved neurological function through the multivariate analysis.

At present, the optimal timing of surgery is still controversial for patients with thoracic Pott's deformity. From the perspective of deformity, some authors [19] have suggested that when tuberculous lesions cause kyphosis to develop to more than 50 degrees, the deformity should be surgically corrected to restore sagittal balance. Jain [20] reported that total vertebral body disease, the treatment of refractory diseases, severe kyphosis, the development of neurological deficits, and a lack of improvement or deterioration are surgical indications for spinal tuberculosis. Based on our data, we suggest the following recommendations. (1) For patients with severe Pott's deformity presenting with neurological symptoms, conservative treatment is ineffective. When MRI images show that the spinal cord is epidurally compressed with spinal edema, myelitis, or myelomalacia, it is necessary to perform surgical decompression as soon as possible. (2) For patients without neurological symptoms, a spinal cord sagittal diameter ratio greater than 47% or a spinal cord angle less than 95° indicated that the local spinal cord was severely stretched. Thus, decompression should be considered to avoid the progression of irreversible neurological symptoms.

There were several limitations to our study. First, this was a single-center retrospective study. A multicenter prospective study with more patients is desirable. In addition, only patients with thoracic kyphosis were included in this study. The thoracic cord is relatively smaller than the thoracolumbar spinal canal [21]. Therefore, with a varied ratio of cord to canal diameter, the threshold values of the spinal cord angle or the ratio of sagittal diameter of the spinal cord may be different.

## 5. Conclusion

In this series of patients with thoracic Pott's deformity undergoing 3-column osteotomies, the spinal cord sagittal diameter ratio and spinal cord angle were predictive of patients developing late-onset neurological deficits. The identification of accurate radiological risk factors can help to determine the surgical timing and to improve the safety and outcomes when performing complex spinal corrections.

## Figures and Tables

**Figure 1:** A 60-year-old male patient suffered from rapid deterioration of neurological symptoms with AIS grade C. (a) Clinical images. (b) Plain radiographs showing angular kyphosis of the upper thoracic region of the spine.

**Figure 2:** Radiological measurement of the patient in Figure 1. (a) The left panel shows the measurement of the spinal cord angle (SCA). (b, A) Sagittal diameter (SD) of the spinal cord at maximum compression; B and C represent SD of the spinal cord one level above or below the site of maximum compression, respectively. Average SD of the spinal cord (D) = (B + C)/2. Spinal cord sagittal diameter ratio (SDR) = (D − A)/D∗100%. (c, A) Spinal cord cross-sectional area (CSA) at maximum compression. B and C represent spinal cord CSA one level above or below the site of maximum compression, respectively. Average CSA of the spinal cord (D) = (B + C)/2. Spinal cord cross − sectional area ratio (CSAR) = (D − A)/D∗100%.

**Figure 3:** A 45-year-old female with spinal tuberculosis presented with 96.8° of kyphosis (a, AIS grade E). (b) CT revealed fusion of T11 and T12 vertebrae. (c) T2-weighted MRI showed tortuous spinal cord in the kyphotic region. SDR was 23.4%. SCA was 127.7°. CSAR was 13.4%. SDR: spinal cord sagittal diameter ratio; SCA: spinal cord angle; CSAR: spinal cord cross-sectional area ratio.

**Figure 4:** A 63-year-old male with spinal tuberculosis presented with 158.5° of kyphosis (a). (b) Preoperative photograph showed obvious stoop (AIS grade B). The patients suffered from delayed paraplegia. (c) CT revealed destruction and fusion of multiple vertebrae from T7 to L1. (d) T2-weighted MRI showed compressed spinal cord in the kyphotic region. SCA was 79.2°. (e) SDR was 64.3%. (f–h) CSAR was 48.3%. (i) MVCR surgical procedure was carried out to resect the vertebrae of T8-12, with posterior pedicle screw fixation and fusion. SDR: spinal cord sagittal diameter ratio; SCA: spinal cord angle; CSAR: spinal cord cross-sectional area ratio.

**Table 1:** Demographic characteristics of patients.

Patient characteristics	Value
Age	45.9 ± 15.8
Gender^∗^	
Male	52 (67)
Female	26 (33)
Duration of kyphosis	32.4 ± 12.6
Anti-TB chemotherapy^∗^	67 (86)
Level of apex^∗^	
T1 to T4	9 (12)
T5 to T8	43 (55)
T9 to T12	26 (33)
Segments involved	6.5 ± 7.6

^∗^The values are given as the number of patients, with the percentage in parentheses.

**Table 2:** Patient AIS grade at first present and final assessment.

AIS grade	Asymptomatic group	Symptomatic group	
		Initial assessment^∗^	Final assessment^∗^
A	0	3 (5)	2 (3)
B	0	8 (13)	5 (8)
C	0	19 (32)	14 (23)
D	0	30 (50)	24 (40)
E	18	0 (0)	15 (25)

^∗^The values are given as the number of patients, with the percentage in parentheses.

**Table 3:** AIS grade conversion from preoperative evaluation to final assessment^∗^.

Initial AIS grade	Final AIS grade				
	A	B	C	D	E
A	2	1	0	0	0
B	0	4	2	2	0
C	0	0	12	5	2
D	0	0	0	17	13

^∗^Data were based on 60 patients from the symptomatic group.

**Table 4:** Quantitative measures and interrater reliability.

	Value^∗^	Interrater reliability^#^
Spinal cord cross-sectional area ratio (%)	45.23 ± 25.67	0.93 (0.89 to 0.97)
Spinal cord sagittal diameter ratio (%)	47.10 ± 15.53	0.94 (0.91 to 0.97)
Spinal cord angle (°)	75.19 ± 19.00	0.89 (0.82 to 0.94)

^∗^The values are given as the mean and the standard deviation. ^#^The values are given as the intraclass correlation coefficient, with the 95% CI in parentheses.

**Table 5:** Imaging measurements of the two groups of patients.

	Asymptomatic group	Symptomatic group	*p* value
Spinal cord cross-sectional area ratio (%)	43.77 ± 13.56	47.65 ± 19.32	0.43
Spinal cord sagittal diameter ratio (%)	40.23 ± 13.25	67.45 ± 12.44	<0.01
Spinal cord angle (°)	109.43 ± 21.35	86.45 ± 17.54	<0.01
Preoperative sagittal Cobb angle (°)	97.34 ± 22.18	105.32 ± 25.42	0.23
Postoperative sagittal Cobb angle (°)	-	45.28 ± 30.23	-
S-DAR (°)	20.13 ± 6.49	24.20 ± 9.86	0.10
Segments involved	5.30 ± 7.86	5.72 ± 8.43	0.85
Spinal cord signal change	6	23	0.79
Levers of apex	9.50 ± 4.52	8.95 ± 6.43	0.74

**Table 6:** The likelihood of spinal cord injury (AIS grades A-D) at the initial and final assessment and showing no improvement.

Variable	Initial assessment		Final assessment		No improvement	
	OR^∗^	*p* value	OR	*p* value	OR	*p* value
Spinal cord cross-sectional area ratio > 45%	5.06 (0.12 to 15.34)	0.13	4.35 (0.24 to 13.17)	0.15	5.29 (0.17 to 18.35)	0.08
Spinal cord sagittal diameter ratio > 47%	12.44 (3.55 to 86.33)	<0.01	8.65 (2.01 to 45.76)	<0.01	10.56 (0.65 to 73.56)	0.76
Spinal cord angle < 95°	7.83 (1.67 to 27.60)	<0.01	5.36 (1.05 to 15.36)	0.02	6.78 (0.64 to 43.17)	0.12
Preoperative sagittal Cobb angle > 104°	1.56 (0.29 to 8.69)	0.45	1.70 (0.32 to 9.43)	0.38	1.49 (0.21 to 8.77)	0.71
Segments involved > 5	3.54 (0.43 to 21.34)	0.38	3.21 (0.55 to 19.37)	0.43	3.67 (0.66 to 24.36)	0.56
Age per year	1.02 (0.05 to 5.38)	0.83	1.13 (0.12 to 7.87)	0.76	1.20 (0.09 to 12.34)	0.54
Time to spinal deformity per year	1.07 (0.65 to 1.23)	0.67	1.21 (0.76 to 1.53)	0.65	1.13 (0.67 to 1.47)	0.29
Spinal cord signal change	1.32 (0.12 to 11.23)	0.33	1.29 (0.04 to 13.20)	0.59	1.38 (0.15 to 14.87)	0.
Kyphosis correction rate > 56%	-	-	-	-	3.23 (0.68 to 23.45)	0.25
Intraoperative neuromonitoring events ≥ 1	-	-	-	-	7.45 (0.56 to 16.75)	0.34
Estimated blood loss > 1745 ml	-	-	-	-	1.56 (0.07 to 13.56)	0.58
Operation time > 325 min	-	-	-	-	2.57 (0.43 to 24.56)	0.46

^∗^The values are given as the OR, with the 95% CI in parentheses.

## Data Availability

The datasets generated during and/or analyzed during the current study are available from the corresponding authors on reasonable request.
